# Developing Machine Learning and Statistical Tools to Evaluate the Accessibility of Public Health Advice on Infectious Diseases among Vulnerable People

**DOI:** 10.1155/2021/1916690

**Published:** 2021-12-17

**Authors:** Wenxiu Xie, Meng Ji, Mengdan Zhao, Kam-Yiu Lam, Chi-Yin Chow, Tianyong Hao

**Affiliations:** ^1^Department of Computer Science, City University of Hong Kong, Hong Kong, China; ^2^School of Languages and Cultures, University of Sydney, Sydney, Australia; ^3^School of Computer Science, South China Normal University, Guangzhou, China

## Abstract

**Background:**

From Ebola, Zika, to the latest COVID-19 pandemic, outbreaks of highly infectious diseases continue to reveal severe consequences of social and health inequalities. People from low socioeconomic and educational backgrounds as well as low health literacy tend to be affected by the uncertainty, complexity, volatility, and progressiveness of public health crises and emergencies. A key lesson that governments have taken from the ongoing coronavirus pandemic is the importance of developing and disseminating highly accessible, actionable, inclusive, coherent public health advice, which represent a critical tool to help people with diverse cultural, educational backgrounds and varying abilities to effectively implement health policies at the grassroots level.

**Objective:**

We aimed to translate the best practices of accessible, inclusive public health advice (purposefully designed for people with low socioeconomic and educational background, health literacy levels, limited English proficiency, and cognitive/functional impairments) on COVID-19 from health authorities in English-speaking multicultural countries (USA, Australia, and UK) to adaptive tools for the evaluation of the accessibility of public health advice in other languages.

**Methods:**

We developed an optimised Bayesian classifier to produce probabilistic prediction of the accessibility of official health advice among vulnerable people including migrants and foreigners living in China. We developed an adaptive statistical formula for the rapid evaluation of the accessibility of health advice among vulnerable people in China.

**Results:**

Our study provides needed research tools to fill in a persistent gap in Chinese public health research on accessible, inclusive communication of infectious diseases' prevention and management. For the probabilistic prediction, using the optimised Bayesian machine learning classifier (GNB), the largest positive likelihood ratio (LR+) 16.685 (95% confidence interval: 4.35, 64.04) was identified when the probability threshold was set at 0.2 (sensitivity: 0.98; specificity: 0.94).

**Conclusion:**

Effective communication of health risks through accessible, inclusive, actionable public advice represents a powerful tool to reduce health inequalities amidst health crises and emergencies. Our study translated the best-practice public health advice developed during the pandemic into intuitive machine learning classifiers for health authorities to develop evidence-based guidelines of accessible health advice. In addition, we developed adaptive statistical tools for frontline health professionals to assess accessibility of public health advice for people from non-English speaking backgrounds.

## 1. Introduction

From Ebola, Zika, to the novel coronavirus pandemic, outbreaks of highly infectious diseases continue to reveal severe consequences of social and health inequalities in both developing and developed countries [1, 2]. Vulnerable people are affected more by the uncertainty, complexity, volatility, and progressiveness of public health crises and emergencies [3, 4]. A key lesson that governments have taken from the ongoing coronavirus pandemic is the importance of developing disseminating highly accessible, inclusive, actionable, coherent public health advice [5–8], which represents a critical tool to help people with diverse cultural, educational backgrounds and varying abilities to effectively implement health policies at the grassroots level. High variability in people's socioeconomic background, education, and health literacy levels, varying intellectual, cognitive abilities, English proficiency, and religious beliefs can cause barriers to access and implement public health advice under health emergencies and crises [9–11]. Increasing inclusiveness and accessibility of health advice recommendations among diverse vulnerable populations has emerged as an important topic in both public health education and domestic and international policy making as a highly cost-effective measure to reduce health inequalities [12–15].

Currently, there is a lack of national or international guidelines around the development of accessible and inclusive public health advice, especially for health emergencies and crises. However, the recent outbreak of coronavirus has prompted national health authorities to develop highly accessible health resources on COVID-19. Most current public-oriented health resources on infectious diseases belong to regular health resources (RHR) requiring higher levels of education, English proficiency, health knowledge, and literacy [16–19]. Typical RHR are resources published by the World Health Organisation which are intended for both general and professional readerships [20–22]. However, the practical accessibility of WHO health resources among the public remains unknown, as the international health organisation recently embarked on surveys to establish evidence of the accessibility of its public health resources [20].

Vulnerable people-oriented (VPO) health resources are known for their significantly improved language understandability, information relevance (minimal distracting details irrelevant to the readers), social inclusiveness (applicability among diverse people), and information actionability [23–25]. They are developed by medical/health professionals with extensive experiences of working firstly with diverse vulnerable populations to ensure the practical usability of VPO. In English-speaking multicultural societies, intralingual health translations and simplified or accessibility-enhanced English resources provide main sources of public health advice and information for diverse vulnerable populations [8, 26–28], although evidence-based guidelines to inform the development of these materials and associated quality control measures are yet to be established and validated.

Increasing amounts of VPO health resources in English, known as easy-to-read or easy read health materials, provide valuable firsthand materials for the development of assessment instruments and techniques to support best practices in the clinic, as well as global health policy making around accessible health recommendation design and social dissemination. The development of language-adaptive evaluation instruments can facilitate evidence-based health policy making by international health authorities. For health policy makers, we developed supervised Bayesian machine learning classifiers, and for frontline health professionals we developed convenient, language-adaptable statistical analysis tools to evaluate the accessibility of public health advice on top infectious diseases, including COVID-19.

It should be noted that the machine learning classifiers and statistical tools that we developed using Chinese health resources can be conveniently and reliably adapted to other languages using low-cost, relatively easy-to-obtain natural language annotation tools. In doing so, our study provides practical and useful tools for clinical and health professionals working directly with vulnerable people. The intuitive Bayesian probabilistic evaluation tool that we developed will help advance research-based global accessible health advice design and international benchmarking for the pandemic which continues to spread in many developing countries and any future public health crises that require rapid, effective, and efficient response from governments and health authorities to address the practical needs from diverse vulnerable populations and help minimise the environmental and health impacts on them.

## 2. Methods

### 2.1. Collection and Translation of Regular and Vulnerable People-Oriented Health Resources

We collected two sets of stylistically distinct public health advice on the prevention and self-management of infectious diseases. Regular health resources (RHR) (202) were selected from the website of the World Health Organisation (WHO). **Vulnerable People-Oriented** (VPO) materials (91), especially public health advice on COVID-19, were collected from websites of health authorities, including Centers for Disease Control and Prevention (CDC), Australian Ministry of Health and Public Health England. These resources were easily recognisable due to being labelled clearly as easy-to-read public health advice and instructions on COVID-19. As an international health authority, WHO provides verified professional translations of original English resources. Since our study was to develop assessment tools to evaluate accessibility of public health advice in Chinese, Chinese translations of regular WHO health advice on infectious diseases were collected. VPO resources collected from sources of CDC, the Australian Ministry of Health and Public Health, England, were translated into Chinese using forward and backward translation recommended by the WHO [29–31].

### 2.2. Morphological-Lexical-Structural (MLS) Features

The Chinese translations of RHR and VPO were annotated using Chinese Readability Index Explorer (CRIE) [32, 33]. CRIE annotation provided 26 morphological-lexical-structural (MLS) features and 46 part-of-speech (POS) features (72 in total) of the annotated Chinese texts for our machine learning classifier development. MLS included average sentence number per paragraph, type token ratio (TTR), low-stroke characters (1–10 strokes), middle-stroke characters (11–20 strokes), high-stroke characters (21 or above), average strokes per character, 2-character words, 3-character words, average words per sentences, ratio of noun phrases, normalised frequency of noun phrases, average number of idioms per sentence, content words (verbs, nouns, adverbs, and adjectives), adverbs of negation, sentences with complex semantic (polysemous) categories, density of content words, average logarithmic frequency of content words, pronouns, personal pronouns, conjunctions, positive conjunctions, negative conjunctions, and difficult words ratio. These MLS features were studied extensively in Chinese readability research.

### 2.3. Parts of Speech (POS) Features

A POS tagging system developed by Academia Sinica as one of the most comprehensive automatic analysers of Chinese was applied. The POS features collected included nonpredicate adjective (A), coordinate conjunction (Caa), conjunctions (Cab), conjunctions (Cba), correlative conjunctions (Cbb), adverbs (D), nominal/adverbial/complement markers (DE), adverbial noun-modifiers (Da), adverbs of degree before verbs (Dfa), adverbs of degree after verbs (Dfb), tense markers (Di), sentential adverbs (Dk), interjections (I), common nouns (Na), proper nouns (Nb), geographical names (Nc), location names (Ncd), time adverbs (Nd), attributive adjuncts (Nep), modifiers of quantitative measures (Nes), quantities (Neu), measure words (Nf), post-positions (Ng), pronouns (Nh), prepositions (P), Be verbs (SHI), auxiliary words (T), intransitive predicates (VA), causative verbs (VAC), transitive verbs placed after objects (VB), transitive verbs (VC), verbs placed before locations (VCL), predicates used with both direct and indirect objects (VD), action verbs as sentence objects (VE), action verbs as predicate objects (VF), classification verbs (VG), modifiers of verbs and nouns (VH), causative modifiers (VHC), adjectives or past particles placed after objects (VI), transitive verbs to describe states (VJ), mental states and processes (VK), causative predicates (VL), and have verbs (V_2).

### 2.4. Statistical Analysis

Table 1 shows that, among the 72 natural language features (26 MLS, 46 POS), statistically significant differences (*p* < 0.05 of nonparametric Mann-Whitney U tests) between regular health resources (RHR) and vulnerable people-oriented (VPO) health resources were present in 88.9% of the entire feature set: 96.15% (25/26) of morphological-lexical-structural (MLS) features and 84.78% (39/46) of part-of-speech (POS) features. In addition to 2-sided *p* values, we computed Hedges' *g* [34] as corrected Cohen's d (1, 36, and 37) and 95% confidence interval of the effect size estimates. We also provided common language effect sizes (CLES), also known as probability of superiority [35–37]. In our study, CLES allowed an intuitive interpretation of the likelihood of the mean of a certain natural language feature randomly selected from VPO as higher than the mean of that feature in RHR on infectious diseases. We calculated Hedges' *g* and CLES alongside commonly reported *p* values for two purposes: first, this was to help us interpret the result of automatic feature selection using Bayesian machine learning classifiers (Gaussian Naïve Bayes selected due to the presence of normally distributed continuous variables as features); second, this facilitated the determination of sample sizes for follow-up studies or the comparison of effects across studies.

The following formula shows the corrected effect size or Hedges' *g*:

(1) $$\begin{array}{c} \text{Hedges}{}^{\prime }\;g_{s}=\text{Cohen}{}^{\prime }s\;d_{s}\times \left(1-\frac{3}{4\left(n_{1}+n_{2}\right)-9}\right). \end{array}$$

The following formula shows common language effect size (CLES):

(2) $$\begin{array}{c} Z=\frac{\left|x_{1}-x_{2}\right|}{\sqrt{\left(SD_{1}^{2}+SD_{2}^{2}/2\right)}}. \end{array}$$

When computing effect sizes (Hedges' *g*_*s*_) and associated probabilities of superiority (CLES), we used RER as reference class. As a result, positive values indicated that features were statistically higher in more difficult regular health resources; and negative values suggested that features were prevalent in highly accessible, vulnerable people-oriented public health advice. MLS features which had large (absolute value larger than 1), corrected effect sizes, Hedges' *g*_*s*_, and CLES included the following: average sentences per paragraph (VPO: M = 0.601, SD = 0.345; RHR: M = 3.316, SD = 1.163, *p* < 0.001, Hedges' *g*_*s*_ = 2.588, 95% CI [2.301, 2.874], and CLES = 0.966); type token ratio (TTR) (VPO: M = 0.461, SD = 0.119; RHR: M = 0.623, SD = 0.079, *p* < 0.000, Hedges' *g*_*s*_ = 1.828, 95% CI [1.568, 2.088], and CLES = 0.902); frequency of difficult words (VPO: M = 141.813, SD = 96.381; RHR: M = 70.872, SD = 35.986, *p* < 0.001, Hedges' *g*_*s*_ = −1.311, 95% CI [−1.558, −1.065], and CLES = 0.823); single sentences (VPO: M = 0.883, SD = 0.114; RHR: M = 0.460, SD = 0.191, *p* < 0.001, Hedges' *g*_*s*_ = −2.376, 95% CI [−2.655, −2.098], and CLES = 0.954); pronouns (VPO: M = 41.692, SD = 35.043; RHR: M = 1.469, SD = 1.652, *p* < 0.001, Hedges' *g*_*s*_ = −2.530, 95% CI [−2.814, −2.245], and CLES = 0.963); personal pronouns (VPO: M = 37.868, SD = 31.838; RHR: M = 0.705, SD = 1.139, *p* < 0.001, Hedges' *g*_*s*_ = −2.577, 95% CI [−2.864, −2.291], and CLES = 0.966); low-stroke characters (VPO: M = 641.593, SD = 444.264; RHR: M = 284.707, SD = 140.930, *p* < 0.001, Hedges' *g*_*s*_ = −1.507, 95% CI [-1.758, −1.256], and CLES = 0.857); 2-character words (VPO: M = 256.637, SD = 176.783; RHR: M = 114.341, SD = 56.262, *p* < 0.001, Hedges' *g*_*s*_ = −1.509, 95% CI [−1.76, −1.258], and CLES = 0.857); and average logarithmic frequency of content words (VPO: M = 1.738, SD = 0.169; RHR: M = 1.337, SD = 0.183, *p* < 0.001, Hedges' *g*_*s*_ = −2.225, 95% CI [−2.498, −1.952], and CLES = 0.942).

Part of speech (POS) features which had large (absolute value larger than 1), corrected effect sizes, Hedges' *g*_*s*_, and CLES included the following: Nh (pronouns) (VPO: M = 41.692, SD = 35.043; RHR: M = 1.469, SD = 1.652, *p* < 0.000, Hedges' *g*_*s*_ = −2.530, 95% CI [−2.814, −2.245], and CLES = 0.963); VF (action verbs as predicate objects) (VPO: M = 4.198, SD = 3.964; RHR: M = 0.222, SD = 0.629, *p* < 0.001, Hedges' *g*_*s*_ = −2.119, 95% CI [−2.388, −1.849], and CLES = 0.933); VA (intransitive predicates) (VPO: M = 11.659, SD = 10.140; RHR: M = 2.088, SD = 2.214, *p* < 0.000, Hedges' *g*_*s*_ = −1.919, 95% CI [−2.181, −1.656], and CLES = 0.913); VK (mental states and processes) (VPO: M = 9.736, SD = 7.688; RHR: M = 2.293, SD = 2.086, *p* < 0.000, Hedges' *g*_*s*_ = −1.889, 95% CI [−2.151, −1.627], and CLES = 0.909); D (adverbs) (VPO: M = 44.110, SD = 31.491; RHR: M = 14.489, SD = 8.247, *p* < 0.001, Hedges' *g*_*s*_ = −1.849, 95% CI [−2.11, −1.589], and CLES = 0.905); VC (transitive verbs) (VPO: M = 48.791, SD = 35.985; RHR: M = 14.759, SD = 10.551, *p* < 0.001, Hedges' *g*_*s*_ = −1.812, 95% CI [−2.071, −1.552], and CLES = 0.900); Ncd (location names) (VPO: M = 6.747, SD = 5.960; RHR: M = 1.869, SD = 1.933, *p* < 0.001, Hedges' *g*_*s*_ = −1.526, 95% CI [−1.777, −1.274], and CLES = 0.860); P (prepositions) (VPO: M = 22.571, SD = 16.570; RHR: M = 9.330, SD = 6.188, *p* < 0.001, Hedges' *g*_*s*_ = −1.424, 95% CI [−1.672, −1.175], and CLES = 0.843); and V_2 (have) (VPO: M = 4.560, SD = 5.879; RHR: M = 1.128, SD = 1.214, *p* < 0.001, Hedges' *g*_*s*_ = −1.197, 95% CI [−1.44, −0.953], and CLES = 0.801).

### 2.5. Gaussian Naïve Bayes

Gaussian Naïve Bayes (GNB) is a variant of Naïve Bayes which is supervised machine learning classification algorithm based on the Bayes theorem [38–42]. Various strengths of GNB are its convenience, computation speed (suitability for making real time prediction), scalability, generalisability with small data like most Bayesian machine learning classifiers, and flexibility with continuous and discrete features. In our study, the size of the training (205) and testing data (88) was relatively small. Bayesian machine learning classifiers like GNB, relevance vector machine (RVM), and multinominal Naïve Bayes (MNB) are more suitable, as they are unlikely to overfit small datasets. Furthermore, the two sets of public health resources that we collected, regular and vulnerable people-oriented sets, contained continuous features and their distributions in the Chinese translations of regular health resources followed Gaussian normal distribution (Table 2, Figure 1). As a result, GNB was selected as the most suitable machine learning classifier in our study to ensure the generalisability and reliability of the classifiers.

### 2.6. Training and Testing Machine Learning Classifiers

To train machine learning classifiers for automatic information accessibility evaluation, the total number of RHR used was 202 and the total number of VPO used was 91. Next, 73.3% (148) of RHR and 62.6% (57) of VPO were used as the training data and the remaining texts (54 RHR and 34 VPO) were used as testing data. We applied 5-fold cross-validation with the training data to produce the mean and standard deviation of area of curve (AUC) of the GNB classifier. Review of the model performance was on the remaining 30% test data in terms of AUC, accuracy, sensitivity, specificity, and macro F1 (Table 3).

### 2.7. Classifier Optimisation

High dimensional features can reduce the performance of machine learning classifiers due to the forced inclusion of irrelevant parameters in the model. To counter the issue of classifier underperformance caused by the presence of redundant features, we applied different classifier optimisation techniques to reduce the original features collected. First, we applied integral optimisation by selecting the optimised feature set from the combined MLS and POS features (72 in total). This led to a combinedly optimised feature set of 6 features (around 8% of the original total features): average sentences per paragraph (ASPP) (*p* < 0.000, Hedges' *g*_*s*_ = 2.588, 95% CI [2.301, 2.874], and CLES = 0.966), personal pronouns (*p* < 0.001, Hedges' *g*_*s*_ = −2.577, 95% CI [−2.864, −2.291], and CLES = 0.966), Di (tense markers) (*p* < 0.001, Hedges' *g*_*s*_ = −1.003, 95% CI [−1.243, −0.763], and CLES = 0.761), Nd (time adverbs) (*p*=0.002, Hedges' *g*_*s*_ = −0.418, 95% CI [−0.65, −0.186], and CLES = 0.616), VF (action verbs as predicate objects) (*p* < 0.001, Hedges' *g*_*s*_ = −2.119, 95% CI [−2.388, −1.849], and CLES = 0.933), and V_2 (have verbs) (*p* < 0.001, Hedges' *g*_*s*_ = −1.197, 95% CI [−1.44, −0.953], and CLES = 0.801).

These optimised features were also those with the most significant statistical differences (indicated by *p* values, corrected effect size Hedges' *g*, common language effect sizes CLES) between regular and vulnerable people-oriented health resources (Table 1). Next, we applied feature optimisation in the two sets of MLS (26) and POS (46) features separately. This led to an optimised MLS feature set of 2 features only (7.7% of the total MLS features): ASPP and ALFCW (*p* < 0.001, Hedges' *g*_*s*_ = −2.225, 95% CI [−2.498, −1.952], and CLES = 0.942). The optimised POS feature set of 8 features (17.4% of the total POS features): A (nonpredicate adjectives) (*p* < 0.000, Hedges' *g*_*s*_ = −0.023, 95% CI [−0.254, 0.207], and CLES = 0.507), Cbb (correlative conjunctions) (*p* < 0.001, Hedges' *g*_*s*_ = −1.022, 95% CI [−1.263, −0.782], and CLES = 0.765), Dfa (adverbs of degree before verbs) (*p* < 0.001, Hedges' *g*_*o*_ = −0.797, 95% CI [−1.033, −0.561], and CLES = 0.713), Nd (time adverbs) (see above), Ng (postpositions) (*p* < 0.001, Hedges' *g*_*s*_ = −1.090, 95% CI [−1.331, −0.848], and CLES = 0.780), Nh (pronouns) (*p* < 0.001, Hedges' *g*_*s*_ = −2.530, 95% CI [−2.814, −2.245], and CLES = 0.963), VCL (verbs placed before locations) (*p* < 0.001, Hedges' *g*_*s*_ = −1.656, 95% CI [−1.911, −1.401], and CLES = 0.879), and VHC (causative modifiers) (*p* < 0.001, Hedges' *g*_*s*_ = 0.649, 95% CI [0.415, 0.884], and CLES = 0.677). For both integral and parallel classifier optimisations, we used backforward feature elimination known as recursive feature elimination (RFE) with support vector machine as base estimator. Maximal validation accuracy/minimal classification errors were used as the feature optimisation criteria (Table 4 and Figure 2).

## 3. Results

Table 3 shows the performance of GNB classifiers using different feature sets. Overall, Bayesian classifiers using optimised features outperformed those using original, larger feature sets. For example, on the testing data, the integrally optimised GNB with 2 MLS and 6 POS features achieved a higher AUC (0.993), sensitivity (0.963), specificity (0.9118), and accuracy (0.940) than the classifier using the full feature set which had AUC (0.940), sensitivity (0.944), specificity (0.8824), and accuracy (0.921). The separately optimised POS feature set (8 POS features) achieved a higher AUC (0.968), sensitivity (1.0), specificity (0.8824), and accuracy (0.955) than the original POS feature set (46 POS features) (AUC = 0.852, sensitivity = 0.889, specificity = 0.7941, and accuracy = 0.852). After comparing the 3 optimised feature sets: MLS/POS jointly optimised (6), MLS optimised (2), and POS optimised (8), we added the 2 sets of separately optimised features of 2 MLS features (ASPP, ALFCW) and 8 POS features (A, Cbb, Dfa, Nd, Ng, Nh, VCL, and VHC) together and further refined the feature set to 2 features only: ALFCW and Nh (pronouns) using the same backward elimination RFE_SVM procedure. This resulted in a highly simplified model (model 8) which achieved largely comparable performance to the best-performing model, the one which integrated the 2 separately optimised features (model 7). Optimised model 8 achieved higher specificity (1.0) than the model 7 (0.8824), which indicated better detection of public health resources and advice suitable for use under health emergencies and crises for maximal social accessibility.

### 3.1. Bayesian Probabilistic Outputs

The outputs of Bayesian machine learning classifiers are in the form of a probability of belonging to the regular public health advice training data. In our study, for the best-performing classifier (model 8: refined MLS and POS separately optimised: 2 features: ALFCW and Nh), average mean output (probability) was 0.9557 (SD = 0.152; range: 0.02, 1; 95% CI: 0.915, 0.996) for regular public health resources and 0.022 (SD = 0.069; range: 0, 0.28; 95% CI: −0.00118, 0.04518) for vulnerable people-oriented public health advice. The differences among public health advice on infectious diseases (translated to Chinese) in terms of public accessibility (high: vulnerable people-oriented resources; low: regular resources) were statistically significant (*p* < 0.001, Hedges' *g*_*s*_ = 7.367, 95% CI: 6.197, 8.536, and CLES = 1).  Figure 3 is a histogram which shows the number of regular (restricted accessibility) and vulnerable people-oriented (high accessibility) health pieces of advice that fell into each 10% probability bin based on the GNB outputs. One hundred percent of vulnerable people-oriented health advice was assigned a probability of highly accessible health resource equal to or smaller than 50% (specificity = 1); and 98.15% of regular public resources were assigned a probability of public advice of restricted/low accessibility larger than 50% (sensitivity = 98.15%). Around 2% of regular public health resources were misclassified as highly accessible information and advice for the public.

### 3.2. Thresholds and Positive/Negative Likelihood Ratios (LR+)

Although it is intuitive to use 0.5 as the probability threshold (Figure 3), this is not the case in real life scenarios, because the criterion for a meaningful cut-off depends on the desired pair of sensitivity and specificity or the diagnostic utility of the research instrument. In our study, higher classifier sensitivity is indicative of higher precision with the prediction of regular public health advice (from WHO resources) which have restricted public accessibility; and higher classifier specificity implies increased accuracy with the detection vulnerable people-oriented health advice (from 3 national health authorities) which were designed by experienced health professionals to maximally enhance the language, cognitive accessibility, informational actionability, and communicative effectiveness of these emergency pieces of advice among diverse vulnerable populations with limited education, health literary, socioeconomic abilities, and varying intellectual/cognitive capabilities.

Table 5 shows various probability cut-offs and their associated sensitivity and specificity pairs using the best-performing GNB classifier that we developed using 2 features only (ALFCW: average logarithmic frequency of content words; Nh: pronouns). It shows that when setting the cut-offs lower than 0.1, sensitivity was the highest (0.9815) and specificity was 0.9118. This means that if this machine learning system were used to assist with public health advice design and dissemination, less than 2% of public health advice with restricted accessibility would be misclassified as accessible information and less than 10% of highly accessible materials would be misclassified as ineffective public health advice, potentially increasing the budgetary burden to hire experts to review health resources or extend the timeframe of releasing information to the public. When increasing the threshold from 0.1 to 0.2, sensitivity remained unchanged, and specificity increased. From 0.2 to 0.5, specificity (cost related) remained the same, but sensitivity deceased from 0.98 to 0.96, suggesting that 2% of health public with limited accessibility to vulnerable populations would be misclassified as suitable health advice and information. In high-risk scenarios such as the outbreaks of highly infectious diseases among some of the most deprived communities, this misjudgement in health advice planning can be very costly, as vulnerable people would be given less effective, accessible, and protective health advice and information.

Sensitivity continued to decrease when thresholds raised higher than 0.5, despite the fact that specificity reached 1. Positive likelihood ratio (LR+) (the ratio between sensitivity and false positivity) is another measurement of diagnostic utility. A LR + larger than 10 indicates a very large effect on posttest probability of disease or in the case of our study lack of accessibility of public health advice among some of our most vulnerable communities and people, who need accessible, actionable public health advice most. In our study, using the best-performing Bayesian classifier, the highest LR+ 16.685 (95% CI: 4.35, 64.04) was reached when setting the threshold of probability at 0.2 (sensitivity = 0.982, 95% CI: 0.95, 1; specificity = 0.941, 95% CI: 0.86, 1). This represents the safest (highest sensitivity) and the most cost-effective (lowest budget investment in expert hire) model of machine learning-assisted predictive design of accessible public health advice and information for vulnerable people and populations. We hope that this promising result based on machine learning development using low-cost, relatively easy-to-obtain natural language tools would provide more support for evidence-based, user-oriented policy making around inclusive, accessible public health advice design and communication under both regular and emergency circumstances.

## 4. Discussion

### 4.1. Retrospective Assessment of Accessibility of Public Health Advice in Other Languages

Another major strength of our study was that we translated the best practices of accessible health advice on infectious diseases developed by English health authorities during the pandemic into adaptive analytical instruments (low-cost, fast-to-build machine learning algorithms) that can be used for the retrospective assessment of existing health advice in other languages. This was achieved by translating the English materials that we collected to the Chinese language using the forward and backward translation method recommended by WHO and comprehensively annotated the translations using Chinese natural language processing tools to allow automatic feature engineering and machine learning classifier development. Table 5 and Figure 4 illustrate how probabilistic outputs might assist with decision making among policy makers and health/medical professionals when designing public health advice for vulnerable people and communities speaking Chinese or migrants, foreigners living in China or greater China regions. Next, we adapted the machine learning classifier to a convenient statistical tool which can be effectively used in the clinic by health/medical professionals and educators to assess whether a certain piece of health advice on infectious diseases is accessible to vulnerable people (both Chinese and migrants) with limited education and health literacy or Chinese proficiency while living in Chinese speaking regions. We fitted a binary Logistic Regression (LR) model with the 70% training data collected. The model contained two independent variables which were borrowed from the best-performing classifier: **ALFCW** (average logarithmic frequency of content words) and **Nh** (number of pronouns). The fitted model with the regression coefficients was shown as follows.

The following is the binary regression formula:

(3) $$\begin{array}{c} {\text{score}}_{\text{LR}}=-2.67\times ALFCW-0.663\times Νh+7.536. \end{array}$$

We then used the Sigmoid Function to scale the score_LR_ to the region of [0, 1]:

(4) $$\begin{array}{c} \text{Sigmoid}\left(x\right)=\frac{1}{1+e^{-x}}. \end{array}$$

The following formula shows Chinese health advice accessibility assessment tool (CHAAAT):

(5) $$\begin{array}{c} \text{score}=100\times \text{Sigmoid}\left(-2.67\times ALFCW-0.663\times Nh+7.536\right). \end{array}$$

We examined the performance of the CHAAAT formula on the remaining 30% test data which contained 34 highly accessible COVID-19 prevention resources translated from 3 national health authorities in the USA, Australia, and UK and 54 regular health resources on infectious diseases developed by the WHO for the public. Average mean output (transformed score using the Sigmoid Function) was 5.8958 (SD = 18.128, range: 1.51908E-32, 73.5, and 95% CI: −0.194, 12) for highly accessible, vulnerable people-oriented public health advice and resources and 88.363 (SD = 2.34, range: 12.119, 99.466, and 95% CI: 83.665, 93.062) for regular WHO public health resources with limited accessibility among vulnerable people with low education, limited health literacy, and limited Chinese proficiency such as foreigner migrants or people with cognitive impairments.

Differences between the two sets of test data measured by CHAAAT formula were statistically very significant: *p* < 0.001, Hedges' *g*_*s*_ = 7.248, 95% CI: 6.094, 8.401, and CLES = 1. These effect sizes were comparable to those (*p* < 0.000, Hedges' *g*_*s*_ = 7.367, 95% CI: 6.197, 8.536, and CLES = 1) of probabilistic outputs of the best-performing GNB classifier using the same feature pair: AFLCW and Nh.  Figure 5 shows the number of regular (restricted accessibility) and vulnerable people-oriented (high accessibility) health pieces of advice that fell into each 10-score bin based on the transformed scores computed using the CHAAAT regression formula. Ninety-four percent of vulnerable people-oriented health advice were assigned a transformed score of highly accessible health resource smaller than 50 (specificity = 94.12%) and 96.3% of regular public resources were assigned an indicative score of public advice of restricted/low accessibility equal to or larger than 50 (sensitivity = 96.3%).

Around 4% regular (requiring higher literacy and Chinese proficiency) resources were misclassified as highly accessible information and advice for vulnerable communities and people living in Chinese speaking regions. Since the 4% errors can still result in a costly overestimate of the accessibility or usability of public health advice among vulnerable populations who require highly accessible (simple, actionable, and implementable) public health information and advice, like with machine learning classifiers, we could adjust the thresholds of the CHAAAT formula to obtain the desired sensitivity and specificity pair according to the practical needs in the clinic.  Table 6 shows that, like the threshold of the best-performing GNB classifier, setting the threshold of the transformed score (Formula (5)) to 29.906 will allow the regression calculator to achieve the same sensitivity and specificity as the GNB classifier. According to practical needs for accessible public health advice under different circumstances, further decreasing the threshold will lead to increased sensitivity of the assessment tool, which might be needed when the health risks being communicated are complex, and the vulnerability of the target populations is high.

The design and assessment of population-oriented public health advice are high-stakes activities which require highly precise, reliable research tools to support informed, evidence-based public health policy planning and delivery. Our study showed that valuable experiences gained in the design of accessible public advice as triggered by the coronavirus pandemic can be translated to useful, much-needed research instruments and tools to support the design of public health advice for any future health events or crises. Furthermore, we developed assessment tools adaptable to other languages to facilitate international benchmarking and support global public health policy planning around accessible health risk communication and public engagement. The limitation of our study is that we used Chinese as an illustrating example which is a distinct language from English. However, the underlying techniques and methods that we discussed and demonstrated can be conveniently modified for other languages or writing systems, especially underresourced languages such as African languages and minority languages, as we developed high performing Bayesian machine learning classifiers based on small datasets. For illiterate populations, our methods need further adaptation for the assessment of oral public advice and information.

## Figures and Tables

**Figure 1:** Continuous feature distribution in regular health resources (RHR) translated into Chinese.

**Figure 2:** Recursive feature elimination using SVM as base estimator.

**Figure 3:** Percentage of vulnerable people-oriented (VPO) materials and regular health resources (RHR) assigned by GNB to 10 probability bins.

**Figure 4:** Receiver operating characteristic (ROC) of Gaussian Naïve Bayes classifiers.

**Figure 5:** Percentage of vulnerable people-oriented (VPO) or regular health resources (RHR) assigned by CHAAAT to each 10-score bin.

**Table 1:** Mann-Whitney U test.

MLS features (1–26) POS (27–72)	EHR mean	EHR std.	RHR mean	RHR std.	Asymp. sig. (2-tailed)	Effect size *d*_*Cohen*_ (corrected effect size or Hedges' g)	Common language effect size CLES	95% CI	Mann-Whitney U	Wilcoxon W	Z
Average sentences per paragraph	0.601	0.345	3.316	1.163	0.000	2.588	0.966	2.301 to 2.874	52.00	4238.00	−14.669
TTR	0.461	0.119	0.623	0.079	0.000	1.828	0.902	1.568 to 2.088	4389.00	8575.00	−10.680
Difficult words	141.813	96.381	70.872	35.986	0.000	−1.311	0.823	−1.558 to −1.065	8769.50	70897.50	−6.657
Low-stroke characters	641.593	444.264	284.707	140.930	0.000	−1.507	0.857	-1.758 to−1.256	8108.00	70236.00	−7.264
Middle-stroke characters	120.396	80.348	51.810	27.695	0.000	−1.562	0.865	−1.814 to−1.31	7357.00	69485.00	−7.955
High-stroke characters	0.055	0.229	0.452	1.604	0.005	0.277	0.578	0.045 to 0.508	14144.00	18330.00	−2.815
Average strokes per character	7.677	0.274	7.711	0.342	0.195	0.103	0.529	−0.127 to 0.334	14604.00	18790.00	−1.297
2-character words	256.637	176.783	114.341	56.262	0.000	−1.509	0.857	−1.76 to −1.258	8100.50	70228.50	−7.271
3-character words	13.000	11.824	8.298	6.372	0.008	−0.603	0.665	−0.837 to −0.369	13139.50	75267.50	−2.647
Average words per sentences	11.592	4.963	11.893	1.962	0.018	0.106	0.530	-0.125 to 0.336	13438.00	17624.00	−2.368
Single sentences	0.883	0.114	0.460	0.191	0.000	−2.376	0.954	−2.655 to −2.098	949.00	63077.00	−13.851
Ratio of noun phrases	0.267	0.104	0.415	0.198	0.000	0.810	0.717	0.573 to 1.046	8396.50	12582.50	−6.999
Frequency of noun phrases per 10K	322.369	37.240	314.664	37.002	0.028	−0.208	0.558	−0.439 to 0.023	13620.50	75748.50	−2.200
Average idioms per sentences	0.001	0.004	0.012	0.029	0.004	0.424	0.618	0.192 to 0.656	13969.00	18155.00	−2.894
Content words	392.582	265.421	163.074	80.538	0.000	−1.642	0.877	−1.896 to −1.387	6988.50	69116.50	−8.293
Adverbs of negation	2.758	3.067	0.935	1.228	0.000	−1.032	0.767	−1.272 to −0.792	9522.50	71650.50	−6.283
Sentences with complex semantic categories	25.396	22.039	7.614	4.758	0.000	−1.643	0.877	−1.898 to −1.388	6696.50	68824.50	−8.578
Density of content words	0.828	0.026	0.815	0.031	0.000	−0.433	0.620	−0.665 to −0.2	11857.50	73985.50	−3.820
Average logarithmic frequency of content words	1.738	0.169	1.337	0.183	0.000	−2.225	0.942	−2.498 to −1.952	1854.00	63982.00	−13.009
Idioms	0.077	0.268	0.224	0.510	0.009	0.312	0.587	0.081 to 0.544	14168.00	18354.00	−2.623
Pronouns	41.692	35.043	1.469	1.652	0.000	−2.530	0.963	−2.814 to −2.245	620.50	62748.50	−14.398
Personal pronouns	37.868	31.838	0.705	1.139	0.000	−2.577	0.966	−2.864 to −2.291	326.00	62454.00	−15.334
Conjunctions	18.967	16.440	11.520	6.407	0.001	−0.795	0.713	−1.031 to −0.558	12507.50	74635.50	−3.228
Positive conjunctions	16.824	14.159	9.000	5.193	0.000	−0.991	0.758	−1.23 to -0.751	10808.00	72936.00	−4.795
Negative conjunctions	0.846	1.584	1.440	1.393	0.000	0.414	0.615	0.182 to 0.646	10710.50	14896.50	−5.070
Difficult words ratio	30.384	5.724	35.847	8.175	0.000	0.706	0.691	0.471 to 0.941	9400.50	13586.50	−6.077
A	3.099	3.774	3.026	2.969	0.236	−0.023	0.507	−0.254 to 0.207	14740.50	18926.50	−1.184
VI	0.143	0.485	0.159	0.424	0.348	0.037	0.510	−0.194 to 0.267	15418.50	19604.50	−0.938
Dk	0.011	0.105	0.017	0.130	0.680	0.048	0.514	−0.183 to 0.278	15919.00	20105.00	−0.413
VG	2.154	2.454	2.054	1.919	0.505	−0.049	0.514	−0.28 to 0.181	15305.00	19491.00	-0.666
Nv	9.967	10.390	9.290	6.711	0.083	−0.089	0.525	−0.32 to 0.142	14132.00	18318.00	−1.734
Neqb	0.033	0.180	0.057	0.277	0.590	0.092	0.526	−0.138 to 0.323	15810.00	19996.00	−0.539
Cab	0.121	0.390	0.398	0.799	0.000	0.377	0.605	0.145 to 0.609	13151.00	17337.00	−3.534
I	0.033	0.180	0.000	0.000	0.001	−0.406	0.613	−0.638 to −0.174	15488.00	77616.00	−3.414
VAC	0.154	0.392	0.048	0.215	0.001	−0.406	0.613	−0.638 to −0.174	14493.00	76621.00	−3.214
Nd	4.253	7.872	2.298	3.408	0.002	−0.418	0.616	-0.65 to −0.186	12764.50	74892.50	−3.050
Nb	1.451	2.423	0.739	1.420	0.000	−0.425	0.618	−0.657 to −0.193	12369.50	74497.50	−3.789
Dfb	0.066	0.291	0.003	0.053	0.000	−0.451	0.625	−0.683 to −0.219	15181.00	77309.00	−3.831
Neu	4.505	6.339	2.395	3.209	0.001	−0.521	0.644	−0.754 to −0.288	12438.00	74566.00	−3.347
VJ	10.011	8.836	6.455	5.125	0.000	−0.586	0.661	−0.82 to −0.352	11896.00	74024.00	−3.797
VL	2.912	2.946	1.710	1.741	0.001	−0.588	0.661	−0.821 to −0.354	12457.00	74585.00	−3.343
Cba	0.110	0.379	0.003	0.053	0.000	−0.602	0.665	−0.836 to −0.369	14652.50	76780.50	−5.125
Caa	12.846	11.117	8.705	5.150	0.103	−0.608	0.666	−0.842 to −0.374	14244.50	76372.50	−1.631
VB	0.912	1.488	0.321	0.722	0.000	−0.635	0.673	−0.869 to −0.401	12839.50	74967.50	−3.789
VHC	0.527	1.089	1.705	1.958	0.000	0.649	0.677	0.415 to 0.884	9100.00	13286.00	−6.641
Da	0.516	1.058	0.125	0.348	0.000	−0.686	0.686	−0.921 to −0.451	12813.00	74941.00	-4.647
Nes	2.033	2.100	0.960	1.278	0.000	−0.723	0.696	−0.959 to -0.488	10783.50	72911.50	−5.088
Dfa	3.473	3.854	1.608	1.752	0.000	−0.797	0.713	−1.033 to −0.561	10952.00	73080.00	−4.769
VH	22.154	15.913	13.767	8.222	0.000	−0.817	0.718	−1.053 to −0.58	11401.00	73529.00	−4.243
Nf	7.418	8.071	3.094	3.956	0.000	−0.852	0.727	−1.089 to −0.615	9110.50	71238.50	−6.401
Nc	7.780	7.781	2.688	5.303	0.000	−0.864	0.729	−1.101 to −0.627	8121.00	70249.00	−7.430
Nep	3.527	4.388	1.327	1.653	0.000	−0.890	0.736	−1.128 to −0.653	12279.50	74407.50	−3.559
T	1.165	1.662	0.261	0.649	0.000	−0.953	0.750	−1.192 to −0.715	10192.00	72320.00	−6.926
Di	2.901	3.169	0.912	1.538	0.000	−1.003	0.761	−1.243 to −0.763	9200.50	71328.50	−6.755
SHI	4.396	4.942	1.676	1.709	0.000	−1.006	0.762	−1.246 to −0.766	10776.00	72904.00	−4.917
VD	1.703	2.355	0.375	0.861	0.000	−1.012	0.763	−1.252 to −0.772	9587.50	71715.50	−7.241
Cbb	5.890	6.402	2.415	2.001	0.000	−1.022	0.765	−1.263 to −0.782	10325.50	72453.50	−5.297
Neqa	6.011	5.997	2.537	2.227	0.000	−1.034	0.768	−1.274 to −0.794	10036.50	72164.50	−5.553
Na	113.209	77.721	64.639	32.606	0.000	−1.065	0.774	−1.306 to −0.824	11326.50	73454.50	−4.308
Ng	6.473	8.048	2.068	1.980	0.000	−1.090	0.780	−1.331 to −0.848	8874.50	71002.50	−6.668
V_2	4.560	5.879	1.128	1.214	0.000	−1.197	0.801	−1.44 to −0.953	9003.50	71131.50	−6.676
VE	7.824	7.207	2.670	2.913	0.000	−1.237	0.809	−1.482 to −0.993	8111.50	70239.50	−7.335
DE	27.396	21.300	11.653	7.618	0.000	−1.336	0.828	−1.583 to −1.09	8606.50	70734.50	−6.816
P	22.571	16.570	9.330	6.188	0.000	−1.424	0.843	−1.672 to −1.175	8358.00	70486.00	−7.045
Ncd	6.747	5.960	1.869	1.933	0.000	−1.526	0.86	−1.777 to −1.274	7167.50	69295.50	−8.263
VCL	5.242	5.730	0.693	1.033	0.000	−1.656	0.879	−1.911 to −1.401	5248.50	67376.50	−10.615
VC	48.791	35.985	14.759	10.551	0.000	−1.812	0.900	−2.071 to −1.552	5672.50	67800.50	−9.506
D	44.110	31.491	14.489	8.247	0.000	−1.849	0.905	−2.11 to −1.589	5603.00	67731.00	−9.573
VK	9.736	7.688	2.293	2.086	0.000	−1.889	0.909	−2.151 to −1.627	5158.50	67286.50	−10.096
VA	11.659	10.140	2.088	2.214	0.000	−1.919	0.913	−2.181 to −1.656	4616.50	66744.50	−10.605
VF	4.198	3.964	0.222	0.629	0.000	−2.119	0.933	−2.388 to −1.849	4026.50	66154.50	−13.780
Nh	41.692	35.043	1.469	1.652	0.000	−2.530	0.963	−2.814 to −2.245	620.50	62748.50	−14.398

**Table 2:** Continuous feature distribution in regular health resources (RHR) translated to Chinese.

Continuous MLS features	Min	Max	Mean	SE.	95% confidence interval for mean		SD.	Skewness	SE.	Kurtosis	SE.
ASPP	0.122	8.857	2.759	0.072	2.617	2.90	1.518	0.145	0.116	−0.194	0.231
DCW	0.691	0.896	0.817	0.001	0.814	0.820	0.030	−0.210	0.116	0.382	0.231
RNP	0.000	1.271	0.385	0.009	0.367	0.403	0.192	0.826	0.116	1.207	0.231
ALFCW	0.808	2.228	1.420	0.012	1.397	1.442	0.242	0.365	0.116	-0.18	0.231
NFNP	200.00	458.33	316.25	1.765	312.78	319.71	37.14	0.268	0.116	0.616	0.231
ASPC	6.505	8.705	7.704	0.016	7.673	7.734	0.329	-0.264	0.116	1.059	0.231

ASPP: average sentences per paragraph; DCW density of content words; RNP: ratio of noun phrases; ALFCW: average logarithmic frequency of content words; NFNP: normalised frequency of noun phrases; ASPC average strokes per character.

**Table 3:** Performance of Gaussian Naïve Bayes (GNB) classifiers with different feature sets.

Model	Techniques	Training (5-fold CV)	Testing				
		AUC mean (SD)	AUC	Accuracy	Macro F1	Sensitivity	Specificity
1	MLS + POS full (69)	0.971 (0.0212)	0.940	0.921	0.992	0.944	0.8824
2	MLS + POS jointly optimised (6)	0.998 (0.0026)	0.993	0.940	0.943	0.963	0.9118
3	MLS full (26 features)	0.997 (0.003)	1.0	0.966	0.963	1.0	0.9118
4	MLS optimised (2 features)	0.998 (0.004)	1.0	0.943	0.938	1.0	0.8529
5	POS full (46 features)	0.959 (0.0238)	0.907	0.852	0.843	0.889	0.7941
6	POS optimised (8 features)	0.982 (0.0166)	0.968	0.955	0.951	1.0	0.8824
7	MLS + POS separately optimised (10)	1.0 (0)	1.0	0.955	0.951	1.0	0.8824
8	Refined MLS + POS separately optimised (2)	0.995 (0.0079)	0.999	0.989	0.988	0.982	1.0

**Table 4:** Criteria of classifier optimisation.

Techniques	Cross-validation accuracy (CVA)	Minimal classification error (MCE) = 1-CVA
Joint optimisation (6)	0.9853	0.0147
Optimised MLS features (2)	0.9902	0.0098
Optimised POS features (8)	0.9854	0.0146

**Table 5:** Thresholds, positive/negative likelihood ratio, and 95% CI of the best-performing GNB classifier on the test data.

Probability thresholds	Sensitivity (95% CI)	Specificity (95% CI)	Positive likelihood ratio (LR+) (95% CI)	Negative likelihood ratio (LR-) (95% CI)
0.1	0.982 (0.95, 1.0)	0.9118 (0.82, 1.0)	11.12 (3.77, 32.79)	0.02031 (0.003, 0.142)
**0.2**	**0.982 (0.95, 1.0)**	**0.941 (0.86, 1.0)**	**16.69 (4.35, 64.04)**	**0.01968 (0.003, 0.137)**
0.5	0.963 (0.91, 1.0)	0.941 (0.86, 1.0)	16.37 (4.26, 62.87)	0.039 (0.010, 0.154)
0.6	0.963 (0.91, 1.0)	1.0 (1.0, 1.0)	Infinity	0.037 (0.010, 0.144)
0.7	0.9444 (0.883, 1.0)	1.0 (1.0, 1.0)	Infinity	0.0556 (0.019, 0.167)
0.9	0.9074 (0.830, 0.985)	1.0 (1.0, 1.0)	Infinity	0.09259 (0.0402, 0.213)
Machine learning classifier: refined GNB classifier (with ALFCW and Nh features)				

**Table 6:** Thresholds of transformed scores of CHAAAT regression formula.

Score thresholds	Sensitivity	Specificity	Score thresholds	Sensitivity	Specificity
1.828	1.000	0.853	64.118	0.926	0.941
7.685	1.000	0.882	66.222	0.907	0.941
16.462	0.981	0.882	68.542	0.889	0.941
25.144	0.981	0.912	70.964	0.870	0.941
**29.906**	**0.981**	**0.941**	72.994	0.870	0.971
43.160	0.963	0.941	73.327	0.852	0.971
59.899	0.944	0.941	76.001	0.852	1.000

## Data Availability

The data that support the findings of this study are available upon request from the corresponding author.

## References

[1] The Lancet (2020). Redefining vulnerability in the era of COVID-19. *The Lancet*.

[2] McBain R. K., Wickett E., Mugunga J. C., Beste J., Konwloh P., Mukherjee J. (2016). The post-ebola baby boom: time to strengthen health systems. *The Lancet*.

[3] Ahmed F., Ahmed N. E., Pissarides C., Stiglitz J. (2020). Why inequality could spread COVID-19. *The Lancet Public Health*.

[4] Saunders M. J., Evans C. A. (2020). COVID-19, tuberculosis and poverty: preventing a perfect storm. *European Respiratory Journal*.

[5] Paakkari L., Okan O. (2020). COVID-19: health literacy is an underestimated problem. *The Lancet Public Health*.

[6] (2020). *Risk Communication and Community Engagement Readiness and Response to Coronavirus Disease (COVID-19)*.

[7] Hu G., Qiu W. (2020). From guidance to practice: promoting risk communication and community engagement for prevention and control of coronavirus disease (COVID‐19) outbreak in China. *Journal of Evidence-Based Medicine*.

[8] Nezafat Maldonado B. M., Collins J., Blundell H. J., Singh L. (2020). Engaging the vulnerable: a rapid review of public health communication aimed at migrants during the COVID-19 pandemic in Europe. *Journal of Migration and Health*.

[9] Teo C. L., Chee M. L., Koh K. H. (2021). COVID-19 awareness, knowledge and perception towards digital health in an urban multi-ethnic Asian population. *Scientific Reports*.

[10] Zarocostas J. (2020). How to fight an infodemic. *Lancet*.

[11] Biancovilli P., Makszin L., Jurberg C. (2021). Misinformation on social networks during the novel coronavirus pandemic: a quali-quantitative case study of Brazil. *BMC Public Health*.

[12] Prem K., Liu Y., Russell T. W. (2020). The effect of control strategies to reduce social mixing on outcomes of the COVID-19 epidemic in Wuhan, China: a modelling study. *The Lancet Public Health*.

[13] May T. (2005). Public communication, risk perception, and the viability of preventive vaccination against communicable diseases. *Bioethics*.

[14] SoleimanvandiAzar N., Irandoost S. F., Ahmadi S. (2021). Explaining the reasons for not maintaining the health guidelines to prevent COVID-19 in high-risk jobs: a qualitative study in Iran. *BMC Public Health*.

[15] Kluge H. H. P., Jakab Z., Bartovic J., D’Anna V., Severoni S. (2020). Refugee and migrant health in the COVID-19 response. *The Lancet*.

[16] Castro-Sánchez E., Spanoudakis E., Holmes A. H. (2015). Readability of ebola information on websites of public health agencies, United States, United Kingdom, Canada, Australia, and Europe. *Emerging Infectious Diseases*.

[17] Mishra V., Dexter J. P. (2020). Comparison of readability of official public health information about COVID-19 on websites of international agencies and the governments of 15 countries. *JAMA Network Open*.

[18] Berland G. K., Elliott M. N., Morales L. S. (2001). Health information on the internet. *JAMA*.

[19] Storino A., Castillo-Angeles M., Watkins A. A. (2016). Assessing the accuracy and readability of online health information for patients with pancreatic cancer. *JAMA Surgery*.

[20] Ennis M., McKay B., Mylan L., Dyke E., Deonandan R. (2016). http://www.who.int/docs/default-source/documents/evaluation/report-evaluation-impact-who-publications.pdf?sfvrsn=577627c5_2.

[21] https://www.who.int/mediacentre/communication-framework.pdf.

[22] Fernández-Díaz E., Iglesias-Sánchez P. P., Jambrino-Maldonado C. (2020). Exploring WHO communication during the COVID 19 pandemic through the WHO website based on W3C guidelines: accessible for All?. *International Journal of Environmental Research Public Health*.

[23] Chinn D. (2020 Mar). An empirical examination of the use of easy read health information in health consultations involving patients with intellectual disabilities. *Journal of Applied Research in Intellectual Disabilities*.

[24] Song P., Karako T. (2020). COVID-19: real-time dissemination of scientific information to fight a public health emergency of international concern. *BioScience Trends*.

[25] Guterman E. L., Braunstein L. Z. (2020). Preprints during the COVID-19 pandemic: public health emergencies and medical literature. *Journal of Hospital Medicine*.

[26] Orcutt M., Patel P., Burns R. (2020). Global call to action for inclusion of migrants and refugees in the COVID-19 response. *The Lancet*.

[27] Zarcadoolas C. (2011). The simplicity complex: exploring simplified health messages in a complex world. *Health Promotion International*.

[28] Zhang J., Wu Y. (2020). Providing multilingual logistics communication in COVID-19 disaster relief. *Multilingua*.

[29] Wild D., Grove A., Martin M. (2005). Principles of good practice for the translation and cultural adaptation process for patient-reported outcomes (PRO) measures: report of the ISPOR task force for translation and cultural adaptation. *Value in Health*.

[30] Tsang S., Royse C., Terkawi A. (2017). Guidelines for developing, translating, and validating a questionnaire in perioperative and pain medicine. *Saudi Journal of Anaesthesia*.

[31] WHO QOL Translation Methodology https://www.who.int/docs/default-source/publishing-policies/whoqol-100-guidelines/translation-methodology.pdf?sfvrsn=74cdb8f5_2.

[32] Li Y., Zhou X., Zhou Y. (2021). Evaluation of the quality and readability of online information about breast cancer in China. *Patient Education and Counseling*.

[33] Sung Y. T., Chang T. H., Lin W. C., Hsieh K. S., Chang K. E. (2016). CRIE: an automated analyzer for Chinese texts. *Behavior Research Methods*.

[34] Lakens D. (2013). Calculating and reporting effect sizes to facilitate cumulative science: a practical primer for t-tests and ANOVAs. *Frontiers in Psychology*.

[35] Liu X. S., Carlson R., Kelley K. (2019). Common language effect size for correlations. *The Journal of General Psychology*.

[36] Rice M. E., Harris G. T. (2005). Comparing effect sizes in follow-up studies: ROC Area, Cohen’s d, and r. *Law and Human Behavior*.

[37] Hanel P. H., Mehler D. M. (2019). Beyond reporting statistical significance: identifying informative effect sizes to improve scientific communication. *Public Understanding of Science*.

[38] John G. H., Langley P. Estimating continuous distributions in bayesian classifiers. https://arxiv.org/abs/1302.4964.

[39] Kamel H., Abdulah D., Al-Tuwaijari J. M. Cancer classification using Gaussian naive bayes algorithm.

[40] Gayathri B. M., Sumathi C. P. (2016). An automated technique using Gaussian naive bayes classifier to classify breast cancer. *International Journal of Computer Applications*.

[41] Yarkoni T., Poldrack R. A., Nichols T. E., Van Essen D. C., Wager T. D. (2011). Large-scale automated synthesis of human functional neuroimaging data. *Nature Methods*.

[42] Huang Y., Li L. Naive bayes classification algorithm based on small sample set.

